The article "Rules of Engagement: Epithelial-Microbe Interactions and Inflammatory Bowel Disease" was published in 2021. Journal: Front Med (Lausanne).

# Rules of Engagement: Epithelial-Microbe Interactions and Inflammatory Bowel Disease

**DOI:** 10.3389/fmed.2021.669913

**Published:** 2021-08-27

**Authors:** Albert E. Jergens, Shadi Parvinroo, Jamie Kopper, Michael J. Wannemuehler

**Affiliations:** ^1^Department of Veterinary Clinical Sciences, College of Veterinary Medicine, Iowa State University, Ames, IA, United States; ^2^Department of Veterinary Microbiology and Preventive Medicine, College of Veterinary Medicine, Iowa State University, Ames, IA, United States

**Keywords:** IBD, microbiota, dog, mouse, intestinal permeability, epithelial barrier

## Abstract

Inflammatory bowel diseases (IBD), including Crohn's disease (CD) and ulcerative colitis (UC), are complex, multifactorial disorders that lead to chronic and relapsing intestinal inflammation. The exact etiology remains unknown, however multiple factors including the environment, genetic, dietary, mucosal immunity, and altered microbiome structure and function play important roles in disease onset and progression. Supporting this notion that the gut microbiota plays a pivotal role in IBD pathogenesis, studies in gnotobiotic mice have shown that mouse models of intestinal inflammation require a microbial community to develop colitis. Additionally, antimicrobial therapy in some IBD patients will temporarily induce remission further demonstrating an association between gut microbes and intestinal inflammation. Finally, a dysfunctional intestinal epithelial barrier is also recognized as a key pathogenic factor in IBD. The intestinal epithelium serves as a barrier between the luminal environment and the mucosal immune system and guards against harmful molecules and microorganisms while being permeable to essential nutrients and solutes. Beneficial (i.e., mutualists) bacteria promote mucosal health by strengthening barrier integrity, increasing local defenses (mucin and IgA production) and inhibiting pro-inflammatory immune responses and apoptosis to promote mucosal homeostasis. In contrast, pathogenic bacteria and pathobionts suppress expression and localization of tight junction proteins, cause dysregulation of apoptosis/proliferation and increase pro-inflammatory signaling that directly damages the intestinal mucosa. This review article will focus on the role of intestinal epithelial cells (IECs) and the luminal environment acting as mediators of barrier function in IBD. We will also share some of our translational observations of interactions between IECs, immune cells, and environmental factors contributing to maintenance of mucosal homeostasis, as it relates to GI inflammation and IBD in different animal models.

## Introduction

The inflammatory bowel diseases (IBD), including Crohn's disease (CD) and ulcerative colitis (UC), are complex, multifactorial inflammatory diseases affecting the gastrointestinal (GI) tract (1, 2). IBD is an immune-mediated disorder comprising two distinct phenotypes having varying clinical, endoscopic, immunologic and histopathologic features (3, 4). Crohn's disease is characterized by patchy, transmural inflammation that primarily affects the terminal ileum but can also involve the small intestine. Ulcerative colitis causes diffuse superficial mucosal ulcerative inflammation restricted to the rectum and colon. The cause for IBD remains unknown but it is likely that genetically susceptible individuals develop an aberrant immune response to their microbiota, leading to chronic inflammation and repetitive injury to the intestines (2). The onset of IBD typically occurs in the second or third decade of life but rising incidence worldwide suggest a prominent role for environmental factors (5).

The article "Rules of Engagement: Epithelial-Microbe Interactions and Inflammatory Bowel Disease" was published in 2021. Journal: Front Med (Lausanne).

The intestinal epithelium is composed of a monolayer of columnar epithelial cells that communicate continually with the luminal microbiota and an underlying network of innate and adaptive immune cells. This mucosal barrier normally prevents the entry of pathogenic microbes and toxins while regulating the absorption of nutrients, electrolytes, and water from the lumen into the systemic circulation (6). There is a growing body of data indicating that dysfunction of the intestinal barrier is a causative factor in the pathogenesis of IBD. For example, numerous IBD genetic risk loci affect pathways active in epithelial cells involved in essential functions such as innate immunity, autophagy and endoplasmic stress (7). Moreover, epithelial barrier dysfunction secondary to chronic inflammation and recurring “flares” is characteristic of IBD (8). During active disease, inflammatory mediators (cytokines/bacterial products) released in the intestinal mucosa progressively damage the epithelium and expose mucosal immune cells to luminal antigens that amplify the inflammatory response (3, 9). Finally, the intestinal epithelium is actively involved in repair mechanisms that promote mucosal healing through re-epithelialization to patch defects and maintain mucosal homeostasis (10, 11). Also contributing to maintenance of the mucosal barrier is the controlled replenishment of intestinal epithelial cell (IEC) subtypes (e.g., columnar cells, goblet cells, enteroendocrine cells and Paneth cells) from LGR5 intestinal stem cells (12). In this review, we will focus on the role of IECs and the luminal environment (including the microbiota) to act as mediators of barrier function in IBD. We will also share some of our translational observations of interactions between IECs, immune cells, and environmental factors (including the gut microbiota) contributing to loss of mucosal homeostasis as it relates to GI inflammation and IBD in different animal models.

The article "Rules of Engagement: Epithelial-Microbe Interactions and Inflammatory Bowel Disease" was published in 2021. Journal: Front Med (Lausanne).

### Intestinal Barrier and Mucosal Homeostasis

#### Structural Components of the Epithelial Barrier

The term *mucosal barrier* was first proposed by Cummings in 2004 and describes the complex structure that separates the luminal environment from the internal milieu (13). The intestinal mucosal barrier is a functional entity consisting of separate but interlinked components, including physical elements (e.g., the underlying vascular endothelium, epithelial cells, and the mucus layer), along with a chemical layer composed of digestive secretions, immune molecules, and cellular products (cytokines, inflammatory mediators, and antimicrobial peptides). Apart from these layers, the microbiota also contributes to barrier integrity along with immune functions and GI motility. The intestinal epithelium is composed of a single layer of columnar cells and different specialized cell subtypes: enterocytes, goblet cells, Paneth cells, enteroendocrine cells and immune cells, including intraepithelial lymphocytes (IELs) and dendritic cells (Table 1; Figure 1) (15). Three types of junctional complexes [tight junctions (TJ), adherens junctions (AJ) and desmosomes] provide mechanical cohesion to these columnar cells and seal the paracellular space to regulate the movement of water ions and small molecules across the intestinal mucosa (16–18).

**Table 1:** Components of the intestinal epithelial barrier and their perturbation in IBD.

**Components**	**Function**	**Known defects**
**Physical Barrier**		
Mucus layer	Adherent and loose layers, contain AMPs and microbiota (loose layer)	Reduced thickness to mucus layer, bacterial biofilm with CD, altered composition to mucus layer
Enterocytes	Digestion, macromolecule transport, secrete β-defensins	Defective defensin production, mucosal ulceration/erosions
Goblet cells	Secrete mucin and trefoil factors	Decreased number of goblet cells
Paneth cells	Secrete α-defensins, Reg3 proteins, lysozyme, BMPs for ISC niche	Reduced antimicrobial activity
Enteroendocrine cells	Produce serotonin and 5-HT; sense microbial metabolites	Altered enteroendocrine secretion
Intercellular junctions	Intercellular transport, regulate barrier function	Altered expression and localization
Intra-epithelial lymphocytes (IELs)	Immune surveillance, cytotoxic activity	Imbalance in IEL cytolytic and regulatory functions
Dendritic cells	Antigen sampling	Increased activation promoting inflammation
Plasma cells	Produce secretory IgA (sIgA), help maintain ISC niche	Increased in number, increased granzyme B and cytotoxic activities
**Chemical Barrier**		
Digestive secretions	Degrade nutrients and bacteria	Altered secretions
Anti-microbial peptides (AMPs)	Bacterial degradation and exclusion	Reduced antimicrobial activity
Cytokines, inflammatory mediators	Promote inflammation	Increased production contributing to repetitive mucosal injury

*BMPs, bone morphogenic proteins; 5-HT, 5 hydroxytryptamin; ISC, intestinal stem cell; CD, Crohn's disease*.

The article "Rules of Engagement: Epithelial-Microbe Interactions and Inflammatory Bowel Disease" was published in 2021. Journal: Front Med (Lausanne).

**Figure 1:** Physical and chemical components of the intestinal epithelial barrier. See text for component specifics. With epithelial barrier dysfunction (insert), intestinal permeability increases which allows for antigens and macromolecules (bacteria) to pass into the lamina propria where innate and acquired immune cells reside. From: (14) with permission.

Tight junctions form the most apical adhesive (JP) and are continuous around the IEC at the border between apical and lateral membrane regions (16–18). They function as a semi-permeable paracellular barrier that move ions and solutes through the intercellular space while excluding luminal antigens, bacteria and their toxins. Within TJ complexes are integral transmembrane proteins, occludin and members of the claudin family, that link adjacent cells to the actin cytoskeleton to regulate paracellular permeability (16). Claudins represent a family of TJ proteins that regulate the movement of water and electrolytes through sealing molecules and pores. Experimental studies indicate that differential claudin expression (either up- or down-regulation) is associated with impaired barrier function (19, 20). The important TJ adapter proteins, zonulin occludens (ZO) -1, -2 and -3, connect the cytoskeleton to the transmembrane TJ proteins. Underneath the TJs are the AJs that are important for cell-to-cell signaling and epithelial restitution, while desmosomes provide structural stability between the IECs (16, 21). Summarizing, the intestinal epithelium maintains its selective barrier function through the formation of complex protein-protein networks that mechanically link adjacent IECs to selectively seal the intercellular space.

The expression pattern of JPs is tightly regulated and varies by intestinal compartment (small vs. large intestines), villus/crypt location, and cell membrane location (apical, lateral or basolateral). The expression of AJ and TJ proteins is a dynamic process that is steadfastly regulated by phosphorylation causing both beneficial and harmful consequences (22–24). For example, phosphorylation can either promote TJ protein formation to enhance barrier function or alternatively it can disrupt and redistribute TJ and AJ proteins to increase intestinal permeability (25, 26).

The article "Rules of Engagement: Epithelial-Microbe Interactions and Inflammatory Bowel Disease" was published in 2021. Journal: Front Med (Lausanne).

The human intestinal epithelium constantly renews itself every 4–5 days under normal homeostasis, with the pace of renewal increasing following damage. Regulating this process are pluri-potential stem cells that give rise to all GI epithelial cell lineages and can generate whole intestinal crypts (12). At the tips of villi and along the epithelia of the colon, mature cells undergo apoptosis and are normally shed into the GI lumen. Intestinal stem cells (ISCs that express LGR5) can differentiate into four specialized cell types, including columnar cells (enterocytes and colonocytes), goblet cells, enteroendocrine cells and Paneth cells (the latter cell type found only in the small intestine) (15). Columnar cells are the most abundant epithelial cell found in the small and large intestines and are involved in absorption. Goblet cells produce and secrete mucin (e.g., mucin-2) which covers the surface of the intestinal epithelium. Antimicrobial peptides and lysozyme further fortify the antimicrobial properties of the mucus compartment to promote antigen elimination. Paneth cells produce lysozyme and several antimicrobial peptides to protect against microbial infection including α-defensins and Reg3 proteins (27, 28). They also reside adjacent to ISCs and provide the necessary growth factor (e.g., Wnt, EGF or Notch) signals to the ISCs and constitutes the stem cell's niche (12). Epithelial cells secrete β-defensins in response to sensing of microbes by their pattern recognition as either commensal bacteria or pathogens. Secretory immunoglobulin A (sIgA) is produced by plasma cells to mediate protection at mucosal surfaces by binding bacteria and viruses to prevent their attachment to or invasion of IECs (i.e., immune exclusion) (29). Finally, the resident bacteria provide a deterrent to microbial invasion and maintenance of mucosal homeostasis through competitive exclusion, nutrient utilization, niche localization and their production of bacteriocins (30).

#### Intestinal Barrier Permeability Pathways

The intestinal epithelium serves as the primary compartment of the mucosal barrier and uses both transcellular and paracellular mechanisms to transport substances from the lumen into the lamina propria. The transcellular pathway primarily transports nutrients and compounds having high molecular weight (>600 Da) by means of endocytosis or carrier-dependent transport systems. The protein complexes interconnecting enterocytes (i.e., TJ, AJ, and desmosomes) are dynamic key modulators that allow for the paracellular transport of water, small solutes and electrolytes between enterocytes while restricting the passage of microbes and large molecules (31, 32). Since paracellular transportation occurs through the space between cells, it is less selective as compared to the transcellular pathway which is regulated by membrane channels. Taken together, these two pathways selectively regulate the degree of permeability for substances having different physiochemical properties, such as variable size and ionic charge, into the lamina propria. Any impairment in the integrity or function of these transporting routes increases intestinal permeability which is implicated in the pathogenesis of several GI and extra-GI diseases (i.e., having local or systemic manifestations) such as IBD, celiac disease, type I diabetes, and emotional stress (33, 34).

The article "Rules of Engagement: Epithelial-Microbe Interactions and Inflammatory Bowel Disease" was published in 2021. Journal: Front Med (Lausanne).

The gut microbiome, which contains 10^14^ bacteria and 100-fold more genes than the entire human genome, has a pivotal role in development of the host immune system and metabolism (35). A well-balanced symbiotic relationship between the gut microbiota and the host is required for maintenance of mucosal homeostasis. There are approximately 1,000 different bacterial species within five dominant phyla (i.e., *Bacteroidetes, Firmicutes, Actinobacteria, Proteobacteria, and Verrucomicrobia)* that comprise the healthy human fecal microbiota (36). In contrast, the core gut bacteria in the feces of specific pathogen free (SPF) mice contains 37 genera (37). In this group, *Anaerostipes* spp were present in all mice and are an important butyrate producing bacterial species contributing to mucosal barrier integrity. Another murine microbe with high prevalence is *Parabacteroides* spp which are important in stimulating host immunity. The other dominant murine bacteria include carbohydrate-utilizing and lactate and/or acetate-producing microbes such as *Bifidobacterium* spp and *Lactobacillus* spp. These observations suggest that the composition of a core microbiome within a species is essential for maintaining gut homeostasis and are reflective of overall host health to a variable extent.

#### Methods to Investigate the Intestinal Epithelial Barrier

The intestinal epithelial barrier remains selectively permeable if its integrity is not compromised. Following mucosal barrier disruption, intestinal permeability increases and delivers phlogistic dietary and/or microbial products to the mucosal immune system which provoke host responses. Therefore, the normally tolerogenic crosstalk between the host and the microbiota becomes perturbed resulting in the generation of an overactive immune response. Overtime, this continuous immune stimulation gives rise to intestinal inflammation which triggers the onset of chronic GI disease, such as IBD. Longitudinal studies in patients with IBD indicate that altered intestinal permeability precedes relapse of CD, suggesting a pathogenic role for barrier dysfunction in IBD as well as an indicator of impending symptoms (38). There are several methods for assessment of intestinal permeability via administration of oral probes, *in vitro* or tissue measures, and endoscopic evaluation of the intestinal epithelial barrier (mucosa) in humans (Table 2) (14, 21).

The article "Rules of Engagement: Epithelial-Microbe Interactions and Inflammatory Bowel Disease" was published in 2021. Journal: Front Med (Lausanne).

**Table 2:** General means for assessment of intestinal permeability in humans and animals.

**Method**	**Human**	**Animal**	**Material needed**	**Comments**
**Orally administered probes**				
Lactulose/mannitol	X	X	Urine	Time consuming
FITC-dextran		X	Serum	Time consuming
51Cr-EDTA	X	X	Urine	Time consuming; radiation hazard
***In vitro*** **/tissue measures**				
Ussing chamber	X	X	Biopsies	Invasive; requires specialized equipment
TEER	X	X	Biopsies	Invasive; requires specialized equipment
Histology	X	X	Biopsies	Invasive; permits specialized testing (IHC, confocal microscopy) for TJP expression
Scanning electron microscopy	X	X	Biopsies	Invasive; specialized fixative; expensive
DNA/RNA extraction	X	X	Biopsies	Invasive; permits qPCR for TJP expression
**Biomarkers**				
LAL assay (LPS)	X	X	Plasma	May have technical limitations
Citrulline	X	X	Plasma	Reliability in the dog is questioned
FABP	X	X	Plasma	ELISA performed on plasma or urine
**Endoscopic measures**				
Confocal endomicroscopy	X	X^*^		^*^As performed in dogs; specialized equipment; expensive
Endoscopic mucosal impedance	X			Directly measures duodenal impedance; specialized equipment; expensive

*Modified from references 20 and 38; TEER, trans-epithelial electrical resistance; LPS, lipopolysaccharide; FABP, fatty acid binding protein; IHC, immunohistochemistry; TJP, tight junction protein*.

* *denote that this intervention is only used in dogs*.

Our own work using a defined microbiota [colonized with the altered Schaedler flora (ASF)] mouse model shows that healthy ASF mice have increased intestinal permeability as compared to conventionally reared (CONV) mice. Using RNA *in situ* hybridization, we provide evidence that greater concentrations of bacteria (EUB probe) and/or their products translocate into the cecal lamina propria vs. bacterial products that translocate in CONV mice (Figure 2). Furthermore, ASF mice demonstrated greater IgG antibody response against members of their resident microbiota when compared to the antibody response directed against these same bacteria in CONV mice (unpublished observations). Our findings are in accordance with previously published data confirming that mice harboring a less diverse gut microbiota have an altered mucosal barrier and increased intestinal permeability (40).

The article "Rules of Engagement: Epithelial-Microbe Interactions and Inflammatory Bowel Disease" was published in 2021. Journal: Front Med (Lausanne).

**Figure 2:** RNA *in situ* hybridization for total bacteria (EUB probe) in murine cecal tissue specimens. Red staining indicates the presence of bacteria and/or their products within the cecal lamina propria of ASF colonized mice **(A)** and conventional mice **(B)**. From: Parvinroo et al. (39) with permission.

### Microbiota Alterations in IBD

#### Observations in Human IBD

Abundant clinical studies indicate a dysfunctional interaction between the gut microbiota and the host response in the onset and pathogenesis of IBD. Increased risk of IBD is associated with changes in composition/structure of the intestinal microbiota or genetic predisposition that impairs normal microbial sensing, both of which can cause altered host-microbe interactions (2, 3, 41–48). CD and UC are not considered single gene disorders, as over 240 susceptibility and IBD risk loci have now been identified (49, 50). Twin studies showed that while there is a genetic basis for IBD, it is not inherited in a simple Mendelian fashion (51). Genetic linkage analysis studies have identified nine disease loci, five of which meet the most stringent linkage analysis criteria, the remaining of which were at least suggestive (49). Mutations in several genes responsible for innate immune sensing of the intestinal microbiota, including NOD2/CARD15, IL-23R and ATG16L1, can also lead to increased risk for IBD (52–54). CARD15/NOD2 was the first IBD susceptibility gene that was identified emphasizing the importance of mucosal-microbial disturbances in the pathogenesis of IBD (53). CARD15 encodes an intracellular protein expressed in multiple immune system components including Paneth cells, monocytes, tissue macrophages and intestinal epithelial cells (52, 55–57). In Paneth cells, NOD2 mediates activation of NF-κB that leads to the induction of defensins. With NOD2 mutations in CD, selective α-defensin production is attenuated which predisposes intestinal epithelial cells to microbial infection (58). Additionally, two autophagy genes, ATG16L1 and IRGM—both of which have roles in the processing of microbial antigens as part of the innate immune system—were identified as susceptibility genes (54, 59). Polymorphisms in these genes promote deranged innate immune responses leading to persistent intracellular bacterial infection that promote the development of IBD. IBD has also been linked to IL-10 deficiencies in humans. In the study by Glocker et al., investigators found that mutations in either IL10RA or IL10RB are associated with severe early onset enterocolitis in children (60). In a separate study, investigators reported NOD2 mutations in patients with IBD that were linked to inhibition of IL-10 in human monocytes (61).

The article "Rules of Engagement: Epithelial-Microbe Interactions and Inflammatory Bowel Disease" was published in 2021. Journal: Front Med (Lausanne).

The host microbiota plays an important role in the pathogenesis of IBD as evidenced by numerous clinical studies. Antibiotic use, both in early childhood and in adults, has been associated with increased risk for development of IBD (62). Moreover, the risk for IBD increases following an episode of infectious gastroenteritis (63). There are other observations implicating the microbiota including reports that mucosal inflammation is localized to gut segments with the greatest bacterial loads (2, 42). Furthermore, antibiotic treatment may be effective in a subset of IBD patients (post-surgical, CD and in pouchitis patients). Antibiotics have been used with varying degrees of success and longevity of response in patients with CD having luminal disease, fistulizing disease, and secondary septic complications such as post-operative infections (64). Results from large scale clinical trials and meta-analyses have been mixed with some analyses finding mild to moderate benefits in disease activity scores (65, 66) and others finding no benefit (67). Furthermore, probiotics and fecal microbiota transplant (in UC patients) may induce or maintain remission in some IBD patients (68–70).

Importantly, many studies have shown consistent alterations in microbial communities characterized by reduced microbial diversity in patients with IBD compared to controls (41, 71). The fecal microbiota of both CD and UC patients contains a depletion of Bacteroidetes and Firmicutes phyla (in particular *Clostridium* spp), which are the dominant normal fecal microbiota, and an increased abundance in Proteobacteria (42, 45, 72). Moreover, a metagenomic analysis of microbiomes demonstrated 25% fewer mucosal microbial genes from IBD patients compared with the microbiomes of healthy controls, suggesting that lower microbial diversity is present and contributing to disease (73). Several studies have found decreased abundance of *Faecalibacterium prausnitzii* (74), a major butyrate producing bacteria in the gut, and an increase in sulfate-reducing bacteria (SRB) which cause decreased expression of epithelial TJPs to increase intestinal permeability in IBD (75).

Still other studies have focused on the role of the mucosal microbiota that is different than the fecal microbiota between controls and patients with IBD. Using fluorescence *in situ* hybridization, high concentrations of bacteria were shown adherent to the epithelium of IBD patients as a thick biofilm, mainly composed of *Bacteroides fragilis* (43). In one seminal study, a depletion of Lactospiraceae and Bacteroidetes but increased abundance of Proteobacteria and Actinobacter were present in colonic biopsy specimens from both CD and UC patients, relative to control tissue samples (45). The distribution of operational taxonomic units (OTUs) was associated with disease state but not anatomy (small vs. large intestine) or gross pathology. Furthermore, the microbiome collected in multiple GI locations from a large cohort of treatment naïve patients with new-onset CD found an increased abundance of Enterobacteriaceae, Pasteurellacaea, Veillonellaceae and Fusobacteriaceae and a reciprocal decrease of Erysipelotrichales, Bacteroidales and Clostridiales in pediatric IBD samples as compared to controls (45). These changes also correlated with disease status, that is, inflammation had a significant impact on microbial composition. Since several of the underrepresented bacterial phyla in IBD patients are butyrate-producing microbes, depletion of these organisms might reduce butyrate production, which is an important energy source for colonic epithelial cells and may enhance epithelial barrier integrity and mediate GI immune responses (42). Loss of significant quantities of these bacteria that provide key metabolic products (i.e., short chain fatty acids) to the host could exacerbate some forms of IBD (76–78).

The article "Rules of Engagement: Epithelial-Microbe Interactions and Inflammatory Bowel Disease" was published in 2021. Journal: Front Med (Lausanne).

Pathobionts, such as adherent-invasive *Escherichia coli* (AIEC), are present within the mucosa in 21–62% of patients with ileal CD and 0–19% of healthy individuals (79, 80). Dysbiosis is associated with increased levels of oxygen in the intestinal lumen (81), possibly due to increased intestinal permeability and/or mucosal inflammation (82). In the inflamed gut, increased colonic oxygen levels restrict obligate anaerobic populations (e.g., Firmicutes) and increase the abundance of facultative anaerobes, including members of the family Enterobacteriaceae (83). Patients with CD have specific NOD2 variants that lead to defective innate sensing, autophagy, and immune responsiveness to CD-associated AIEC (7, 84). The adhesion molecule CEACAM6 is over expressed in ileal CD patients which also makes individuals more susceptible to mucosal colonization by AIEC (85). AIEC pathobionts strongly adhere to and invade IECs inducing robust pro-inflammatory cytokine secretion (e.g., IFN-γ, TNF-α) which causes direct damage to the intestinal barrier and promotes inflammation. Once within the ileal mucosa, AIECs can reside and replicate within macrophages, leading to an increased pro-inflammatory response (86). In contrast, AIEC colonization does not occur in colonic CD and the lack of AIEC mucosal translocation in UC patients would suggest that *E. coli* does not play a primary role in UC pathogenesis (87).

The article "Rules of Engagement: Epithelial-Microbe Interactions and Inflammatory Bowel Disease" was published in 2021. Journal: Front Med (Lausanne).

#### Observations in Murine Models of Intestinal Inflammation

Most different mouse models support a role for the microbiota in experimental intestinal inflammation. Early studies in mice treated with dextran sodium sulfate (DSS), a chemical irritant that disrupts the colonic intestinal epithelial barrier to contribute to the development of colitis, reported significant increases in intestinal *Bacteroidaceae* and *Clostridium* spp, in particular *Bacteroides distasonis* and *Clostridium ramosum*, in both acute and chronic colitis DSS models (88). In another study, increased numbers of colonic mucin-degrading *Akkermansia muciniphila* and Enterobacteriaceae were correlated to disease activity in DSS-treated mice resembling UC (89). Interleukin-10 knockout (IL-10^−/−^) mice develop spontaneous colitis that is entirely dependent on gut bacteria (90), and where colonic inflammation is attenuated when treated with antibiotics before disease onset (91) or is eliminated altogether in mice housed in a germ free environment (92). Animal models have also shown that intestinal inflammation is transferable through the intestinal microbiota. Germ-free IL-10^−/−^ mice colonized by the intestinal microbiota of IBD patients exhibit increased colitis as compared to mice colonized with the intestinal microbiota derived from healthy human controls (93). In IL-10^−/−^ mice, loss of regulatory IL-10 secretion results in intolerance to their intestinal microbiota, unbalanced pro-inflammatory responses contributing to mucosal barrier disruption, and the development of spontaneous colitis.

The administration of broad or narrow spectrum antibiotics shows different therapeutic activities in various regions of the colon in SPF colonized IL-10^−/−^ mice. Narrow spectrum antibiotics, such as ciprofloxacin or metronidazole, prevented cecal and colonic inflammation in IL-10^−/−^ mice following SPF colonization. Ciprofloxacin was most effective in treating cecal inflammation by reducing aerobic bacteria, including, *E. coli* and *E. faecalis*; whereasmetronidazole was superior in reducing colitis and eliminated anaerobic bacteria (e.g., *Bacteroides* spp) in both the cecum and colon (94). Importantly, while ciprofloxacin and metronidazole prevented the induction of typhlocolitis in IL-10^−/−^ SPF-colonized mice, these antibiotics had little effect after the onset of intestinal inflammation. In contrast, the broad-spectrum combination antibiotic vancomycin-imipenem decreased total luminal bacteria and prevented and treated both cecal and colonic inflammation. Taken together, these studies demonstrate that gut bacteria have differing inflammatory roles with some species initiating onset of intestinal inflammation while other microbe subsets drive chronic colitis (95).

The article "Rules of Engagement: Epithelial-Microbe Interactions and Inflammatory Bowel Disease" was published in 2021. Journal: Front Med (Lausanne).

Additional evidence supporting the role of the microbiota in colitis development is provided by studies using transfer animal models of colitis induced by deficiency of T-bet in innate immune cells. T-bet is a transcription factor that plays a crucial role in development of Th1 cells and in the regulation of innate and adaptive immunity (96). In certain murine models, loss of T-bet in mice lacking B and T cells (*T-bet*^−/−^/*RAG-1*^−/−^) results in transmissible colitis in conventionally raised wild-type mice by co-housing, presumably caused by microbiota transmission (97). In similar fashion, *Casp3/11*-deficient mice, which are normally protected against DSS-induced colitis, lose this protection and become more sensitive to DSS on co-housing with WT mice (98).

Specific pathogenic bacteria have been associated with the development of intestinal inflammation in murine models. *Proteus mirabilis* and *Klebsiella pneumoniae* correlate with colitis in *T-bet*^−/−^/*Rag2*^−/−^ mice, a mouse model resembling UC (97). Different *Helicobacter* spp, including infection with *H. hepaticus* and *H. bilis* or exposure to their antigens, trigger IBD-like disease in susceptible mice. For example, *H. hepaticus* induces chronic colitis in SPF-housed IL-10^−/−^ mice accompanied by increased expression of pro-inflammatory biomarkers IFN-γ, TNF-α and nitric oxide (99). In a separate study, the combination of *H. hepaticus* infection and CD45RB high CD41 T-cell reconstitution resulted in marked disease expression in severe combined immunodeficiency (*SCID*) mice similar to that observed in human IBD (100). Still other experiments employing targeted infection with *H. hepaticus* were able to produce colitis and sometimes colonic tumors in different mouse strains having defects in immune function and/or regulation (101). Our group has previously shown that defined microbiota [i.e., altered Schaedler flora (ASF)] mice are a useful tool to investigate the impact of specific members of the Proteobacteria (e.g., *E. coli, Helicobacter* spp) on the development of colitis. The induction of typhlocolitis in ASF mice colonized with either *H. bilis* or *Brachyspira hyodysenteriae* was accompanied by induction of ASF-specific antibody (102). Using a “multiple-hit” mouse model of colitis, we have shown that colonization of ASF mice with *H. bilis* increased host susceptibility to onset of severe colitis following low dose (1.5%) DSS administration (i.e., inflammatory trigger) (103). An analysis of the molecular/cellular mechanisms revealed increases in mucosal gene expression involving lymphocyte activation and inflammatory cell chemotaxis, with infiltration of more mucosal immune cells in *H. bilis*-colonized mice prior to DSS treatment vs. DSS treatment alone. A subsequent study with a similar experimental design used microarray analysis to demonstrate differential mucosal gene expression associated with alterations in fatty acid metabolism and detoxification in a time course following *H. bilis* colonization (104). This latter study provided preliminary evidence as to the types of factors or changes in the intestinal mucosa (i.e., alterations in housekeeper genes) that potentially predispose the host to the development of typhlocolitis.

The article "Rules of Engagement: Epithelial-Microbe Interactions and Inflammatory Bowel Disease" was published in 2021. Journal: Front Med (Lausanne).

*Citrobacter rodentium* is an attaching and effacing (non-invasive) bacterial pathogen that primarily causes acute typhlocolitis in mice, except when barrier function is impaired or in animals that are genetically susceptible to inflammation where infection can trigger chronic disease (105). The *C. rodentium* infection model was one of the first mouse models to show that composition of the intestinal microbiota influences susceptibility to infection (106), and that infection can alter the composition and spatial distribution of the resident microbiota post-infection (107). Finally, *Fusobacterium varium* isolated from the colonic mucosa of patients with UC was shown to induce experimental ulcerative colitis in mice (108). Collectively, these experimental studies provide compelling evidence that individual resident species are capable of inducing colitis in susceptible mouse models.

### Novel Animal Model Observations Implicating Epithelial Barrier Dysfunction in IBD

Here we relate some of our own work utilizing different animal models to investigate host-microbe interactions mediating chronic intestinal inflammation and the role of the mucosal barrier in these different model systems.

#### The Dog as a Naturally Occurring Model of Chronic Inflammatory Enteropathy

Dogs represent a well-recognized large animal model that naturally develops CIE (also referred to as idiopathic IBD in the veterinary literature), sharing remarkable similarities in etiology, clinical course, histologic lesions and interventional strategies to human IBD (Table 3) (109–116). The obvious advantages of the dog in relation to other common animal models (e.g., rodents, zebra fish) include their large body size, longer life span, and they possess a GI tract of similar size, structure and function to that of humans. Of key importance for translational studies, pet dogs are exposed to the same environmental conditions and even share similar microbiota composition with their owners (117, 118). *Clostridialis, Fusobacteria, Bacteroides* and *Proteobacteria* are the dominant bacteria comprising the healthy canine fecal microbiota (119, 120). Metagenomic analyses in a small cohort of healthy dogs indicate that diet induced changes in microbial composition are not associated with changes in function, and that the fecal microbiota of dogs, mice and humans exhibit a high degree of metabolic and phylogenetic similarity (121). Considering the common microbiota and environmental exposures with humans, there is growing interest in whether similar mechanisms of CIE pathogenesis are shared between species (122).

The article "Rules of Engagement: Epithelial-Microbe Interactions and Inflammatory Bowel Disease" was published in 2021. Journal: Front Med (Lausanne).

**Table 3:** Comparative features of IBD in different animal models.

**Feature**	**Human**	**Dog**	**Rodent**
Genetic basis	Yes	Yes	Engineered
Etiology	Multifactorial and complex	Multifactorial and complex	+/- Multifactorial
Intact immune system	Yes	Yes	+/-
Resident microbiota role	Yes	Yes	Yes
Blood in stool	Yes	Yes	Yes
Diarrhea	Yes	Yes	Yes
Disease activity measures	Clinical indices, biomarkers	Clinical indices, biomarkers	Laboratory markers
Definitive diagnosis	GI mucosal biopsy	GI mucosal biopsy	GI mucosal biopsy
Longitudinal studies	Yes: endoscopy + histology	Yes: endoscopy + histology	Difficult to perform
Primary therapy	Anti-inflammatory drugs	Diet + anti-inflammatory drugs	Anti-inflammatory drugs
Disease heterogeneity	Yes	Yes	Variable
Spontaneous GI flares	Yes	Yes	+/-

*GI, gastrointestinal*.

Certain dog breeds show a predisposition to the development of CIE suggesting a role for host genetics in this disorder. The German shepherd dog, Soft-coated wheaten terrier and Boxer dog/French bulldog have an increased incidence of CIE clinically that has been linked to mutations in innate immune genes, including TLR5, NOD2, and autophagy gene NCF2 (123, 124). Importantly, several of the same breeds (i.e., German shepherds, Boxer/French bulldog) show positive clinical response to administration of antimicrobials, indicating a potential interaction of host susceptibility with the intestinal microbiota in affected dogs. Intestinal biopsies are required to confirm histopathologic inflammation of CIE, with GI endoscopy being the preferred modality to visually inspect the GI mucosa and to acquire targeted biopsy samples. Mucosal lesions of erosions, friability and increased granularity are observed most frequently during endoscopy and correlate best to histopathologic inflammation (Figure 3) (113, 126). Lympho-plasmacytic enteritis of varying severity is the most common type of inflammation often accompanied by changes in mucosal architecture, including villous atrophy/fusion, erosions, ulceration, cryptal changes and/or depletion of colonic goblet cells (Figure 4) (127). Mixed cellular infiltrates are also observed in dogs with epithelial disruption (neutrophils) or in response to invasive mucosal bacteria (macrophages) as occurs with granulomatous colitis.

The article "Rules of Engagement: Epithelial-Microbe Interactions and Inflammatory Bowel Disease" was published in 2021. Journal: Front Med (Lausanne).

**Figure 3:** Endoscopic evidence of intestinal barrier disruption in dogs with CIE. Multifocal erosions are evident within the ileal **(A)** and colonic **(B)** mucosae of different dogs with moderate-to-severe CIE. From: Jergens et al. (125), with permission.

**Figure 4:** Histopathologic evidence of intestinal barrier disruption. Duodenal biopsy showing focally extensive villus erosions covered by neutrophils and cell debris in a dog with CIE. Hematoxylin and eosin (HE) stain. From: (110), with permission.

Like experimental models and human IBD, the intestinal microenvironment is implicated in the development of CIE in dogs. Numerous studies have shown that intestinal inflammation in dogs is accompanied by dysbiosis, where the proportions of *Clostridiales, Fusobacteria, Bacteroidetes* and *Prevotellacea*e are decreased, but the proportion of *Proteobacteria*, including Enterobacteriaceae, is significantly increased compared to healthy dogs (128–130). Mucosal associated *E. coli* are significantly increased with intestinal inflammation of CIE, granulomatous colitis and colorectal cancer (adenocarcinoma) in dogs (114, 131). Granulomatous colitis (GC) is a unique variant of CIE, causing chronic colitis with small volume diarrhea, straining, hematochezia and mucoid feces in predominantly young Boxer dogs. Here, a possible genetic defect in innate immune sensing confers increased susceptibility to *E. coli* invasion of colonic tissues (124). With this immune defect, ineffective respiratory burst impairs the host's ability to eliminate intracellular pathogens, including catalase-positive bacteria. A diagnosis of canine GC is confirmed by mucosal culture and/or fluorescence *in situ* hybridization that identify invasive *E. coli* within the colonic mucosa of affected dogs (Figure 5). In Boxers with GC, long-term remission is observed with antimicrobial eradication of mucosally invasive *E. coli*, suggesting a causal relationship between this bacterial strain and clinical disease (131). Of interest, the observed phylotype of *E. coli* isolated from Boxer dogs with GC bears strong phylogenetic resemblance to the pathobiont *E. coli* strain isolated from CD patients (132).

**Figure 5:** Granulomatous colitis in a 2-year-old English bulldog. **(A)** Endoscopic image of severe colonic granularity (increased texture) involving the descending colon. **(B)** Colonic biopsy from this dog shows clusters (yellow fluorescence) of mucosal associated *E. coli* following fluorescence *in situ* hybridization. From: Jergens et al. (125), with permission.

The article "Rules of Engagement: Epithelial-Microbe Interactions and Inflammatory Bowel Disease" was published in 2021. Journal: Front Med (Lausanne).

The intestinal barrier of dogs with CIE has been investigated to a limited extent. Using duodenal biopsy samples obtained endoscopically from healthy dogs and dogs with CIE, the mucosal expression of claudin-1, -2, -3, -4, -5, -7, and -8; E-cadherin; and β-catenin was determined by immunoblotting and compared between dog groups (133). Results showed no difference in expression of each claudin and β-catenin between healthy dogs and dogs with CIE; while the expression of E-cadherin was reduced in dogs with CIE. Immunofluorescence microscopy (in a subset of CIE dogs) showed decreased intensity of E-cadherin labeling in the apical villi of dogs with CIE. In humans with IBD, a significant correlation between low E-cadherin expression and disease activity has been previously demonstrated (134). In another study, the ratio of IL-1β to IL-1 receptor antagonist (Ra), and the effect of IL-1β on occludin mRNA expression in the duodenal and colonic mucosa were investigated in healthy dogs and dogs with CIE (135). The ratio of IL-1β to IL-1Ra in the colonic mucosa was higher in dogs with CIE vs. healthy dogs. *Ex vivo* cultures of duodenal and colonic biopsies incubated with IL-1β showed reduced expression of occludin mRNA in colonic, but not duodenal, cultures of dogs with CIE. These findings are similar to observations in humans where both occludin mRNA and protein concentrations are reduced in the intestines of CD and UC patients (136). Finally, another study investigated intestinal pro- and active metalloproteinase (MMP) -2 and -9 activities in healthy dogs and dogs with chronic enteropathy (CE) using gelatin zymography. In dogs with CE, there was a greater number of samples positive for pro- and active MMP2 and -9 in the duodenal, ileal and colonic mucosa as compared to healthy dogs (137). Similar findings of elevated matrix metalloproteinases have been reported in dogs with CIE and in humans with IBD (138, 139).

Clinical trials evaluating drug or probiotic therapy have provided indirect evidence on the role of the intestinal barrier in canine CIE. In one trial, the effects of a hydrolyzed diet and oral prednisone on the spatial distribution of mucosal bacteria in dogs with CIE was investigated using FISH (140). Medical therapy was associated with beneficial changes in microbial community structure and enhanced mucosal junctional protein expression in dogs with CIE. The spatial distribution of mucosal bacteria differed with increased numbers of *Bifidobacteria, Faecalibacteria* and *Streptococci* found within adherent mucus of dogs with CIE post-treatment compared to healthy dogs. Using immunohistochemistry (IHC), the expressions of occludin and E-cadherin were increased but zonulin decreased in dogs with CIE following prednisone therapy. Still other studies using multi-strain probiotics for the treatment of canine CIE have shown potential beneficial alterations in junctional proteins that are associated with remission. In one trial, probiotic therapy with VSL#3 was investigated in comparison to combination treatment with prednisone and metronidazole administered continuously to dogs with CIE for 90 days (115). Dogs treated with probiotic showed remission accompanied by changes in beneficial mucosal responses (i.e., increased numbers of FoxP3+ and TGF-β+ cells) and increased mucosal expression of occludin. Another probiotic trial using FISH to investigate the mucosal microbiota showed that remission of dogs with CIE was associated with changes in beneficial bacterial species and up-regulated expression of junctional proteins following 6 weeks of probiotic therapy (141). Both probiotic and standard therapy for CIE (e.g., hydrolyzed diet + oral prednisone) were associated with rapid remission without improvement in histopathologic inflammation. Probiotic therapy was associated with increased expression (IHC) of junction proteins E-cadherin, occludin and zonulin vs. dogs with CIE that received standard therapy (Table 4; Figure 6). Collectively, these observations of increased barrier integrity in dogs receiving glucocorticoid or probiotic therapy for CIE are in broad agreement with studies in UC patients and experimental models of intestinal inflammation (142–145).

The article "Rules of Engagement: Epithelial-Microbe Interactions and Inflammatory Bowel Disease" was published in 2021. Journal: Front Med (Lausanne).

**Table 4:** Probiotic therapy modulates TJP expression in dogs with IBD.

**Colon**	**Claudin-2**	**E-cadherin**	**Occludin**	**Zonulin**
Healthy dogs	91^*^	1,031^*^	1,119^*^	371^*^
Pre-VSL #3 IBD	1,212^∧^	575	131	61
Post-VSL #3 IBD	82	902^∧^	859^∧^	326^∧^

* *P < 0.05 for healthy dogs vs. Pre-VSL #3 IBD dogs*;

∧ *P < 0.05 for Pre-VSL #3 IBD dogs vs. Post-VSL #3 IBD dogs; TJP, tight junction protein. From reference 129*.

**Figure 6:** Immunohistochemistry for expression of tight junction proteins in colonic biopsies of healthy dogs and dogs with CIE before and after probiotic VSL #3 therapy. Healthy dogs generally express increased TJPs as compared to dogs with CIE at diagnosis (pre-VSL #3). A reciprocal increase in TJP expression is observed in dogs with CIE following probiotic treatment (post-VSL #3). **(A)** Claudin expression; **(B)** E-cadherin expression; **(C)** Occludin expression. All images at 20X magnification. From: White et al. (141), with permission.

#### Other Murine Model Observations

*Brachyspira hyodysenteriae* is a Gram-negative anaerobic spirochete and is the causative agent of swine dysentery. The pathogenesis of disease has been studied in mice and pigs and has been shown to rely on the presence of a resident microbiota (146, 147), production of a ß-hemolysin (148), local inflammatory response of the host (149, 150), and recruitment of host inflammatory cells (151). With respect to the need for other resident bacteria, our own research has shown that the colonization of GF mice with *B. hyodysenteriae* failed to induce typhlocolitis in mice, even when mice were observed for 110 days post-colonization. The need for at least one member of the resident microbiota was demonstrated by administering *Bacteroides vulgatus* to GF mice previously colonized with B. hyodysenteriae (i.e., no disease) and typhlocolitis developed within 5 days. This result suggested that the presence of *B. vulgatus* either enhanced the virulence of *B. hyodysenteriae* or induced host innate immune responses that contributed to the resultant inflammatory response. Furthermore, treatment of mice with an antibiotic cocktail to which the spirochete was resistant in their drinking water for 7 days, prior to colonization with *B. hyodysenteriae*, prevented the onset of disease even though the numbers of spirochetes colonizing the cecum and colon were like that of untreated mice with typhlocolitis. In these conventionally reared mice, the role of the resident microbiota was further shown by replacing the antibiotic-containing drinking with normal drinking water and the severe typhlocolitis developed within 15 days. It was shown that the antibiotics significantly reduced the numbers of bacteria in the feces and cecal contents by six to seven log_10_ with the dominant bacterial types remaining being Gram-negative facultative anaerobes and strict anaerobes. One conclusion to be drawn from these results would suggest that the crosstalk between the host and the resident microbiota contributes to disease susceptibility and the severity of the inflammatory response (152, 153).

The article "Rules of Engagement: Epithelial-Microbe Interactions and Inflammatory Bowel Disease" was published in 2021. Journal: Front Med (Lausanne).

It has also been shown that disease caused by *B. hyodysenteriae* can be inhibited by treating mice orally with an extract (i.e., hypoxoside) from *Hypoxis hemerocallidea* corm (also known as *Hypoxis rooperi*, African Potato). Beginning seven days prior to challenge, the oral administration of hypoxoside did not prevent the colonization of *B. hyodysenteriae*, but prevented the onset of typhlocolitis as evidenced by the lack of inflammatory cell infiltration, absence of crypt hyperplasia, and reduction in the expression of cytokine-specific genes regulated by NF-kB activation (149). As with the administration of antibiotics mentioned above, the administration of hypoxoside prevented disease and expression of TNF-α-specific mRNA when treatment began at least 7 days prior to colonization with *B. byodysenteriae*. The need to initiate treatment 7 days prior to colonization with *B. hyodysenteriae* coincides with the turnover of colonic epithelial cells and suggests that the host inflammatory set-point can be altered in the new epithelial cells by affecting which bacteria are present (i.e., antibiotic use) or by changing the responsiveness of the epithelial cells to phlogistic stimuli (i.e., hypoxoside). In this regard, administration of hypoxoside also inhibited crypt epithelial cell hyperplasia following colonization with *B. hyodysenteriae* (Figure 7). The ability to affect epithelial cell responsiveness was further demonstrated by adding conjugated linoleic acid (CLA) to the diet of pigs prior to colonization with *B. hyodysenteriae*. It has been shown that CLA is a ligand for peroxisome proliferator-activated receptor gamma (PPAR-g) and that the activation of PPAR-g promotes mucosal epithelial health by suppression of inflammation and facilitating metabolic reprogramming (i.e., oxidative phosphorylation) of colonic epithelial cells associated with the use of SCFAs derived from microbial metabolism (150, 154). To further demonstrate that the interaction of *B. hyodysenteriae* with the colonic epithelium-induced inflammatory cell recruitment, mice that were treated with anti-CD18 or anti-CD29 to prevent extravasation of neutrophils from blood failed to develop typhocolitis (151). Using *B. hyodysenteriae* as a model of bacterial induced colitis, these studies have demonstrated that the colonic epithelium in association with the resident microbiota is a key contributor of mucosal health or disease.

**Figure 7:** Immunohistochemical detection of proliferating epithelial cells in mice treated with hypoxoside. Mice were either sham treated orally with sterile drinking water (Control) or hypoxoside (Colonized and treated). The mice treated daily with either saline or hypoxoside (15 mg) beginning 8 days prior to colonization with *Brachyspira hyodysenteriae (B. hyo)*. Mice were necropsied 3 days after colonization. One h prior to necropsy, mice received an IP injection of BrDU. Proliferating epithelial cells were identified by labeling their DNA with anti-BrDU using immunohistochemistry. From: (149), with permission.

In the context of IBD, epithelial barrier function is a critical component of maintaining mucosal homeostasis and tissue health. It has been shown that mice (i.e., mdr1a^−/−^) lacking the multiple drug resistance gene P-glycoprotein 170 (Pg-170) develop spontaneous colitis between 8 and 30 weeks of age associated with epithelial barrier dysfunction. As an efflux pump, Pg-170 is highly expressed in colonic epithelial cells and contributes to the removal of xenobiotics and phlogistic compounds from the cytosol (155). As with many murine models of colitis, GF mdr1a^−/−^ mice do not develop colitis and administration of metronidazole in the drinking water ameliorates the colitis, indicating a role for the resident microbiota in the disease process (156, 157). Like the studies performed using hypoxoside, we have shown that treating mdr1a^−/−^ mice with botanical extracts from either *Prunella vulgaris* or *Hypericum gentianoides* prevented or significantly attenuated colitis in mdr1a^−/−^ mice (158, 159). The reduction in colonic inflammation was consistent with the reduction of NF-kB regulated cytokines and chemokines (e.g., CXCL1, CXCL9, CCL2, CCL20, and TNF-α). In companion studies, we demonstrated that administration of caffeic acid to mice increased the expression to *Cyp4b1* (i.e., cytochrome P450) in the colonic mucosal and ameliorated DSS-induce colitis (160). Analogous to Pg-170, CYP4B1 controls the metabolism of proinflammatory compounds in the GI epithelium and contributes to maintenance of the mucosal barrier. Again, this demonstrates the central role colonic epithelial cells have in the attenuation of mucosal inflammation induced by microbial compounds and in the maintenance of mucosal homeostasis and GI health.

The article "Rules of Engagement: Epithelial-Microbe Interactions and Inflammatory Bowel Disease" was published in 2021. Journal: Front Med (Lausanne).

As IECs are also able to take up antigen and PRR ligands, they contribute to the maintenance of mucosal immunity and intestinal health. The importance of the epithelial response to luminal antigens was elegantly demonstrated by examining the inflammatory response in MyD88^−/−^ mice (161). Initially, the authors had reasoned that since much of the mucosal inflammation associated with IBD was associated with production of pro-inflammatory cytokines; the absence of MyD88 should reduce the severity of disease due to impaired recognition of MAMPs derived from the microbiota. However, these authors demonstrated that the MyD88^−/−^ mice developed more severe colitis than the wild-type counterparts. These observations indicated that there is a cytoprotective aspect to the local inflammatory response that is key to mucosal homeostasis. As mentioned above, we had reported that the administration of anti-CD18 or anti-CD29 attenuated lesion severity in mice colonized with *B. hyodysenteriae*. However, if mice were administered a cocktail containing both anti-CD18 and anti-CD29 or neutrophils were depleted, lesions were more severe than in sham treated mice colonized with *B. hyodysenteriae* (151). Like the MyD88^−/−^ mice, the inability to recruit inflammatory cells resulted in a more severe lesion supporting the importance of epithelial cell responses to inflammatory stimuli, at least in moderation. Similarly, the administration of hypoxoside likely had a beneficial effect in inhibiting the typhlocolitis associated with *B. hyodysenteriae* colonization because it attenuated the local inflammatory responses as opposed to inhibiting that response, thus, retaining the cytoprotective benefit of the residual inflammatory response.

The article "Rules of Engagement: Epithelial-Microbe Interactions and Inflammatory Bowel Disease" was published in 2021. Journal: Front Med (Lausanne).

The role of the epithelial cells to support antigen uptake and maintenance of mucosal tolerance is partially mediated by the induction of regulatory T cells (Tregs) and the secretion of IgA (sIgA) in the the GI lumen. Functionally, one of the features of the sIgA is to provide for immune exclusion which would reduce, but not eliminate, microbial antigen interactions with epithelial cells and underlying immune cells (162). To this end, we evaluated the ability of orally administered serum-derived bovine immunoglobulin (SBI) to inhibit DSS-induced murine colitis (163). The SBI would function to bind to bacterial antigens and reduce the innate and/or adaptive immune activation contributing to colitis. Results demonstrated that mucosal inflammation was significantly reduced, there was a decrease in secretion of pro-inflammatory cytokines and a reduction in intestinal fatty acid binding protein and serum amyloid A. As with the use of botanical extracts, dietary CLA and attenuation of neutrophil recruitment, the use of SBI to reduce mucosal inflammation by lessening the phlogistic potential of luminal content on the mucosa while allowing for the beneficial (i.e., cytoprotective) expression of host inflammatory responsiveness.

## Conclusions

Host-microbe interactions play important roles in maintaining homeostasis of the mucosal epithelial barrier as well as contributing to the development of IBD. The concept that the intestinal epithelium serves as a “translator” between the intestinal microbiota and the immune system seems both logical and plausible (164). Here, the epithelium is responsive to signals from the microbiota by means of pathogen recognition receptors and translates these messages into signals that direct mucosal immune cells. Conversely, IECs receive signals from the underlying immune system and translate them into signals that shape intestinal barrier function and the structure and function of the gut microbiota. Dysregulation of the intestinal barrier is a salient feature of IBD in humans and animal models of inflammation, regardless of species. As such, treatment approaches that aim to support gut barrier function have been identified and are currently under review, including nutritional approaches (avoidance of Western-style diet, precision (FODMAP) diet, prebiotics/fibers]; probiotic approaches (select probiotics, multi-strain probiotics, symbiotic preparations); and drug/other approaches (short chain fatty acids, metformin, fecal microbiota transplantation) (14, 21, 165, 166).

The article "Rules of Engagement: Epithelial-Microbe Interactions and Inflammatory Bowel Disease" was published in 2021. Journal: Front Med (Lausanne).

## Author Contributions

AJ, SP, JK, and MW: review design and input, data/narrative analysis, preparation, and review/editing the manuscript. AJ, SP, and MW: performance of experiments. All authors contributed to the article and approved the submitted version.

## Conflict of Interest

AJ serves as consultant for ExeGi Pharma. The remaining authors declare that the research was conducted in the absence of any commercial or financial relationships that could be construed as a potential conflict of interest.

## Publisher's Note

All claims expressed in this article are solely those of the authors and do not necessarily represent those of their affiliated organizations, or those of the publisher, the editors and the reviewers. Any product that may be evaluated in this article, or claim that may be made by its manufacturer, is not guaranteed or endorsed by the publisher.
